RETRACTED

# Bioinformatics Analysis and Experimental Verification Identify Downregulation of COL27A1 in Poor Segmental Congenital Scoliosis

**DOI:** 10.1155/2022/2616827

**Published:** 2022-02-09

**Authors:** Zongshan Hu, Yanjie Xu, Jie Li, Zezhang Zhu, Yong Qiu, Zhen Liu

**Affiliations:** Division of Spine Surgery, Department of Orthopedic Surgery, Nanjing Drum Tower Hospital, The Affiliated Hospital of Nanjing University Medical School, Nanjing 210008, China

## Abstract

**Background:**

Congenital scoliosis (CS) represents the congenital defect disease, and poor segmental congenital scoliosis (PSCS) represents one of its types. Delayed intervention can result in disability and paralysis. In this study, we would identify the core biomarkers for PSCS progression through bioinformatics analysis combined with experimental verification.

**Methods:**

This work obtained the GSE11854 expression dataset associated with somite formation in the GEO database, which covers data of 13 samples. Thereafter, we utilized the edgeR of the R package to obtain DEGs in this dataset. Then, GO annotation, KEGG analyses, and DO annotation of DEGs were performed by “clusterProfiler” of the R package. This study performed LASSO regression for screening the optimal predicting factors for somite formation. Through RNA sequencing based on peripheral blood samples from healthy donors and PSCS cases, we obtained the RNA expression patterns and screen out DEGs using the R package DESeq2. The present work analyzed COL27A1 expression in PSCS patients by the RT-PCR assay.

**Results:**

A total of 443 genes from the GSE11854 dataset were identified as DEGs, which were involved in BP associated with DNA replication, CC associated with chromosomal region, and MF associated with ATPase activity. These DEGs were primarily enriched in the TGF-*β* signaling pathway and spinal deformity. Further, LASSO regression suggested that 9 DEGs acted as the signature markers for somite formation. We discovered altogether 162 DEGs in PSCS patients, which were involved in BP associated with cardiac myofibril assembly and MF associated with structural constituent of muscle. However, these 162 DEGs were not significantly correlated with any pathways. Finally, COL27A1 was identified as the only intersected gene between the best predictors for somite formation and PSCS-related DEGs, which was significantly downregulated in PSCS patients.

**Conclusion:**

This work sheds novel lights on DEGs related to the PSCS pathogenic mechanism, and COL27A1 is the possible therapeutic target for PSCS. Findings in this work may contribute to developing therapeutic strategies for PSCS.

## 1. Introduction

Congenital scoliosis (CS), a congenital vertebral malformation, is caused by abnormal vertebral body development or poor segmentation during embryonic somatoplasty [1]. In clinical practice, CS is defined as a disorder with an abnormality in vertebral body structure, which further results in a Cobb angle greater than 10 degrees in the spine. The prevalence rate of CS among the population is about 0.5-1.0%. CS can be either an isolated deformity or part of a syndrome with other clinical characteristics [2, 3]. According to previous literature, about 30-60% of CS cases are associated with malformations of other organs such as Alagille syndrome and VACTERL syndrome [4, 5]. Abnormalities in vertebral body structure of CS patients often lead to rapid progression of a scoliosis; besides, they can be complicated by other system dysfunction such as impaired lung function due to the limited thoracic development [6, 7]. Apart from affecting physical health, their presence also poses a significant threat to the mental health of patients, and the subsequent medical examinations and treatments will inevitably increase the financial burden on the families and the society.

RETRACTED

Studies have shown that axonal osteogenesis begins in the embryonic stage and occurs during the gestational weeks in humans. At the end of each body segment, the mature cambium is formed. In other words, the skin, muscle, and bone segments are formed, and later, the dermis, osteoporosis (OP), and axis bone are derived, respectively [8]. Congenital spinal deformity (CSD) takes place during the formation of body segments [9]. CSD can be divided into several types, including disabling hemivertebrae, wedge vertebrae, and ductus vertebrae and segmental deformities, mixed deformities, and subsegmental deformities [10]. Spinal deformities usually occur early in the development of an embryo, namely, during the formation of the perigestational somatoplasty, which is the visceral formation stage. Due to the potential associated pathogenesis, malformations in the neurological, visceral, and other cleavage systems are frequently seen, with the commonly seen malformations including neurological malformations, cardiac malformations, visceral malformations, transposition, urinary malformations, common reproductive malformations, OP, and quadruplasty [11–13]. Generally, the etiological study mainly focuses on two aspects: the environmental effects and the genetic defects. The major environmental aspects are high-risk pregnancy, low oxygen, and vitamin deficiency [11]. In recent years, preliminary research on genes has been conducted at home and abroad, and the existing research results support polygenic hereditary diseases. To be specific, one or more genes may lead to different phenotypes of polygenic hereditary diseases; in addition, changes in gene structure and function can cause susceptibility in the patients, while environmental effects can further complicate gene phenotypes [14]. It is generally accepted that environmental factors play a role by causing genetic mutations and regulating the gene transcription and translation levels.

RETRACTED

Based on recent molecular biological research, alterations of gene expression have critical function in the pathogenesis of CS. Studies have shown that mice with Mesp2 gene knockout suffer from segmented somatic disorder, which causes segmented disorder in the spine [15]. Wallin et al.'s study suggested that mice with PAX1 gene defect exhibited signs of vertebral body and disc loss and ultimately CSD [16]. Generally speaking, TBX-6 is associated with segmented CS, while LMXIA is related to dysplastic CS [17]. These data indicate the differential gene expression in different types of CS. PSCS is a kind of abnormal development of the vertebral column formed during the embryonic period. It is divided into block vertebra and unilateral bony bridge [2]. PSCS accounted for 18%~42% of congenital scoliosis, second only to congenital hemivertebrae deformity [7, 18]. However, among the factors leading to the development of spinal deformity, segmented incomplete vertebral deformity is more harmful than hemivertebrae deformity [5, 11]. At present, surgical treatment of congenital segmental scoliosis in adolescents is seldom reported at home and abroad. Therefore, this study treated one type of CS, PSCS, as the object of the study to screen genes closely related to its progression, so as to obtain new advances in the etiology of PSCS for the prevention, early diagnosis, and treatment of PSCS.

## 2. Materials and Methods

### 2.1. Ethics Statement and Information of Subjects

The present work gained approval from the Ethics Committee of Nanjing Drum Tower Hospital, the Affiliated Hospital of Nanjing University Medical School (2021-194-01). The participants were recruited in Nanjing Drum Tower Hospital, the Affiliated Hospital of Nanjing University Medical School, and voluntarily took part in this work after they were informed of the experimental purpose and process.  Table 1 lists the subject inclusion and exclusion criteria. All the participants were classified into 2 groups, namely, PSCS (*n* = 68) and normal control (*n* = 53) groups. Then, we collected fasting venous blood samples from every participant and preserved them at −80°C for subsequent use.

### 2.2. Blood Specimen Processing

Venous blood samples (5 mL) obtained from PSCS patients and healthy subjects were let stand for a 30-minute period at room temperature (RT). Then, the blood samples were centrifuged at 3000*g*/min and 13500*g*/min for 10 min and 15 min, respectively, at 4°C to obtain the serum samples.

RETRACTED

### 2.3. Total RNA Extraction, Library Construction, and Illumina Sequencing

Total RNA extraction and RNA library construction were conducted. In brief, this study adopted the TRIzol reagent (Invitrogen, Carlsbad, CA, USA) for extracting total RNA; then, a NanoPhotometer spectrophotometer (IMPLEN, CA, USA) was employed to test RNA purity. Moreover, RNA integrity and content were evaluated by using the Agilent 2100 Bioanalyzer (Agilent Technologies, CA, USA) and Qubit 2.0 fluorometer (Life Technologies, CA, USA), separately. Ribosomal RNA (rRNA) was removed by using the Ribo-Zero rRNA Removal Kit (Epicentre, USA). Using the NEBnext ultra RNA library prep kit, rRNA-depleted RNA was used to prepare RNA sequencing (RNA-seq) libraries in line with specific protocols. Afterwards, the Agilent 2100 System (NanoDrop ND-1000) was utilized to determine library quality. Then, real-time quantitative PCR (RT-qPCR) was conducted for accurate quantification. At last, we combined all libraries based on data volume and effective content requirements. The Illumina Hiseq 2000 platform was applied for sequencing.

### 2.4. Quality Control and Mapping

In-house Perl scripts were adopted for raw data processing. To this end, reads that contained contaminants, adaptors, or low-quality reads were removed through cleaning raw data. Besides, we determined N, GC, Q20, and Q30 contents for estimating clean read quality. Subsequently, we aligned clean reads to the reference genome (GRCh37/hg19) by adopting HISTAR2.

### 2.5. Quantitative Analysis of Genes

Cuffdiff (v2.1.1) was employed to calculate transcript FPKM. FPKM is the fragment number per kilobase length in one gene per mapped million fragments, which takes into account the impact of gene length and sequencing depth on the fragment number.

### 2.6. Identification of Differentially Expressed Genes (DEGs)

Firstly, we obtained the GSE11854 dataset in the GEO database (https://www.ncbi.nlm.nih.gov/geo/) to study somite formation-related mRNAs. The expression profile data of the GSE11854 dataset consisted of 1 control group (GSM299435) and 12 experimental groups (GSM299423, GSM299424, GSM299425, GSM299426, GSM299427, GSM299428, GSM299429, GSM299430, GSM299431, GSM299432, GSM299433, and GSM299434). We identified DEGs upon the thresholds of *P* < 0.05 and log | fold change (FC) | >1 using the “edgeR” package in R language.

### 2.7. GO, DO, and KEGG Pathway Analyses of DEGs

According to the previous description, we used the R package ClusterProfiler to determine intersected DEGs based on GO functional annotation with related mRNAs. The GO terms were classified as biological processes (BPs), cellular components (CCs), and molecular functions (MFs). In addition, the R package DOSE was employed for DO annotation analysis to determine gene-disease interactions. By adopting the R package ClusterProfiler, we analyzed KEGG pathways enriched by differentially expressed mRNAs (DEmRNAs) upon the *P* < 0.05 criterion.

RETRACTED

### 2.8. LASSO Regression Analysis

The least absolute shrinkage and selection operator (LASSO) algorithm represents the compression estimation approach, which can construct the penalty function to obtain the refined model; as a result, certain coefficients can be compressed, while some are set to zero. As a result, it contributes to retaining subset shrinkage's advantages; meanwhile, it also represents the biased estimate to process the multicollinearity data. Notably, parameter *λ* controls the adjustment level of complexity of LASSO regression, with a greater *λ* indicating the larger linear model penalty with a greater number of variables. In this way, a model that involves fewer variables can be acquired at last.

The present work established the LASSO regression model using the R package glmnet on the basis of gene expression levels, with disease genesis being a dependent variable (experimental = 1; control = 0) and diverse genes being the independent variables. The model settings are shown as follows: predictive model number, lambda = 1000; type, Gaussian; and LASSO regression standard parameter, alpha = 1.

### 2.9. Quantitative Real-Time PCR (RT-PCR)

This study utilized the TRIzol reagent (Invitrogen, USA) to extract total blood RNA in accordance with specific protocols. By adopting the First Strand cDNA Synthesis Kit (Qiagen, Germany), we prepared cDNA through reverse transcription. Thereafter, the ABI SYBR^®^ Green PCR Master Mix (Applied Biosystems, Foster City, CA) was adopted for the RT-PCR procedure, with GAPDH being the endogenous control. The primer sequences used in this study are shown as follows: COL27A1: GAGGTCCTCACTTCCAGGAG (forward) and AGGACGCTGAACGTCACTAT (reverse), and GAPDH: ACCCAGAAGACTGTGGATGG (forward) and TCAGCTCAGGGATGACCTTG (reverse). The 2^−ΔΔCt^ approach was utilized to determine relative gene expression.

### 2.10. Statistical Analysis

GraphPad Prism (version 8) and R 4.1.1 were utilized for statistical analysis. The Wilcoxon rank-sum test (two-sided), the nonparametric statistical hypothesis test usually adopted to compare between 2 groups, was adopted for data analysis. RT-PCR data were later analyzed by Student's *t*-test, with *P* < 0.05 indicating statistical significance.

RETRACTED

## 3. Results

### 3.1. Identification of DEGs in the Somite Formation-Associated GSE11854 Dataset

We preprocessed and annotated the GSE11854-derived matrix file using the official gene symbol. Later, the R package “edgeR” was employed to identify DEGs upon the thresholds of *P* < 0.05 and FC > 2.0 (logFC > 1.0). At last, we discovered altogether 443 DEGs (Figure 1(a)). In comparison with black plaques, there were 222 upregulated DEGs within red plaques and 221 downregulated DEGs within green plaques (Figure 1(b), Table 2).

### 3.2. Functional Enrichment Analysis of DEGs in the Somite Formation-Associated GSE11854 Dataset

For better investigating biological roles of those 443 discovered DEGs, we conducted functional annotation, as presented in Figure 1(c). According to BP results in GO analysis, there were 47 DEGs associated with DNA replication (adjusted *P* value = 6.77*E* − 27 and *Q* value = 5.90*E* − 27). Meanwhile, based on CC results in GO analysis, there were 33 DEGs associated with the chromosomal region (adjusted *P* value = 9.44*E* − 12 and *Q* value = 8.91*E* − 12), while MF results in GO suggested 28 DEGs associated with ATPase activity (adjusted *P* value = 4.00*E* − 05 and *Q* value = 3.75*E* − 05).

We identified 8 enriched KEGG pathways upon the thresholds of *Q* value < 0.05 and *P* value < 0.05, including the “DNA replication,” “cell cycle,” “cellular senescence,” and “TGF-beta signaling pathway” pathways (Figure 1(d)). At last, based on DO analysis, those 443 DEGs were mainly related to spinal deformity and ovarian cancer (Figure 2(a)). We found that a total of 19 DEGs were closely related to spinal deformity (Figure 2(b)).

### 3.3. LASSO Regression Analysis of Candidate Hub Genes

For observing and predicting whether the identified DEGs affected somite formation, this study established the LASSO regression model using the R package glmnet on the basis of gene levels, so as to estimate the relation of gene levels with disease in an algorithmic manner. Firstly, we chose the suitable model. In Figure 3(a), those 2 dotted lines stand for 2 specific *λ* values (max = 9). Using the prediction model, we identified altogether 9 DEGs as the independent prognostic factors (genes), including ORC6, GALE, CDT1, KIRREL3, CD83, LOC101926996, SHF, COL27A1, and BC034416 (Figure 3(b)). As a result, these prognostic factors were the possible hub genes to predict somite formation.

### 3.4. Identification of DEGs in Patients with PSCS

Using the R package “DESeq2”, we identified PSCS-related DEGs between 3 PSCS patients and 2 healthy subjects based on the abovementioned thresholds. Finally, we discovered 162 DEGs (Figure 4(a)), including 45 with upregulation within red plaques and 117 with downregulation within blue plaques, relative to black plaques (Figure 4(b), Table 3).

RETRACTED

### 3.5. Functional Enrichment Analysis of PSCS-Related DEGs

For better investigating biological roles of those 162 DEGs, this study conducted functional enrichment analysis, as observed from Figure 5(a). According to GO analysis, DEGs were related to BPs and MFs. The BPs in GO showed that circulatory system development and cellular component morphogenesis were significantly associated with DEGs (Figure 5(b)). The MFs in GO revealed that the structural constituent of muscle was significantly related to DEGs (Figure 5(c)). There was no KEGG pathway enriched upon the thresholds of *Q* value < 0.05 and *P* value < 0.05 (Figure 5(d)). On the other hand, the “histidine metabolism,” “cardiac muscle contraction,” “hypertrophic cardiomyopathy (HCM),” “insulin resistance,” “leukocyte transendothelial migration,” and “Apelin signaling pathway” pathways were enriched (*P* value = 0.0086, 0.0325, 0.0332, 0.04, 0.042, and 0.049, respectively, and Figure 5(e) and Table 4).

### 3.6. COL27A1 as the Hub Gene for PSCS Prediction as well as Experimental Validation

As revealed by Venn analysis, COL27A1 was the only overlapping DEG between the LASSO model and the PSCS-associated gene set (Figure 6(a)). For better testing whether these hub genes were important, we chose COL27A1 to conduct RT-PCR validation. As a result, relative to the control group, COL27A1 mRNA expression remarkably decreased in the PSCS group upon the *t*-test (Figure 6(b)).

## 4. Discussion

PSCS is a special type of congenital spinal deformity, which has the most important characteristic of spinal bridge formation without the segmental spine [1, 9, 10]. Bone bridge formation is closely related to genetic factors, genetic abnormalities, abnormal blood vessel development, and transient ischemia at the end of the embryo [4, 5]. Early bone bridge can be cartilaginous with no obvious early symptoms, which leads to the difficulty in diagnosis, and the missed rate of bone bridge on X-ray film is as high as 80.4%. With the application of 3D CT reconstruction techniques, the detection rate of bone bridge is up to 100%, which increases the proportion of segmental disorders that is traditionally considered to be relatively low and tends to exceed that of hemivertebral malformations [2, 19]. Bone bridges can be divided into anterior, anterolateral, posterior, and annular bone bridges according to their position. The progression rate and deformity degree of scoliosis are related to the extent, number, location, and growth potential of bone bridge. Ring bone bridge can form block vertebra and result in obstacle in the symmetrical growth and development of vertebral body segment. In addition, it only manifests as body shortening and loss of intervertebral body activity. The average annual aggravation is no more than 0.5 degrees, and the deformity degree is no more than 20 degrees. Spinal scoliosis deformity caused by unilateral bone bridge formation is more rapid [20]. Due to the formation of two or more intervertebral bones on the one side of the vertebral body, bone fusion induces unbalanced growth and development on both sides of the vertebral body, finally leading to the formation of a segmental spine composed of multiple vertebral bodies. Typically, the shape of the spine is determined by the potential for growth on both sides of the spine and the balance of growth. Generally speaking, the greater segmental span of a single distal segmental bone bridge that affects the growth potential of the side with segmental disturbance will induce the faster progression of spinal deformity and the heavier scoliosis [19, 21]. Thus, the treatment regimen for segmented scoliosis is different from that for other types of spinal deformities.

RETRACTED

During the vertebrate embryonic development, a certain number of temporal structures, called somites, are formed along the front and rear axes of the body. As the embryo continues to develop, each somatic node will differentiate into a bony, dermal, and muscular segment [22]. In this study, only one dataset related to body segments (GSE11854) was collected from the GEO database. Genes can regulate the formation of the somatic ganglion and form synchronous oscillatory expression with the latter. Therefore, Kusumi et al. induced human progenitor fibroblasts and screened genes for the synchronous oscillation with somatic nodes. We identified altogether 9 DEGs as the marker molecules for somatic ganglion formation. Of them, five genes (CD83, LOC101926996, SHF, COL27A1, and BC034416) were synchronously upregulated in the somatic ganglion and four genes (ORC6, GALE, CDT1, and KIRREL3) were significantly downregulated in the somatic ganglion. LOC101926996 and BC034416 are informal and presumptive gene names and may be replaced by more appropriate names in the future. Therefore, subsequent analysis does not consider these two genes. The vertebral column of vertebrates is derived from the somatic nodes. A study will be more accurate when it investigates fewer variables. There are three types of CS, and this group only studied the PSCS type. Thus, we sequenced the blood samples from PSCS patients and obtained 162 DEGs from them. To isolate the hub gene associated with PSCS development, we performed the Wayne analysis of these PSCS-associated DEGs and the nine abovementioned genes that synchronously oscillated with body segments. The results showed that COL27A1 was the only intersected gene. Interestingly, COL27A1 expression increased during somatic nodule formation but significantly decreased in PSCS patients. This suggests that COL27A1 is important for spinal column formation.

RETRACTED

COL27A1, which belongs to the collagen gene family, shows expression within cartilage tissues, such as cartilage [23]. COL27A1 is associated with osteochondral dysplasia, since it contains the rare recessive alleles that can cause bone deformities during embryonic development. COL27A1 is responsible for encoding one proalpha chain in type XXVII collagen, which can join 42 additional genes and integrate their protein products for the formation of 28 or more diverse trimeric collagens [24]. Mouse col27a1 is the most significantly upregulated within cartilaginous tissues of the 14.5-day embryos, such as the spine, rib, and long bone anlage, together with the otic capsule and eye, just like expression levels of genes for type II/XI collagens [25]. During the 19 gestational days, col27a1 showed the most significant upregulation within nasal cartilages, whereas the lowest expression is shown within tooth-forming cells and the gastrointestinal tract [26]. As for human beings, col27a1 was expressed within hand long bone anlage in the 10.8-week embryos; meanwhile, its expression was measured within the trachea as well [24, 26]. In human beings, COL27A1 expression can be detected during the 18-20 gestational weeks within fetal epiphyseal cartilage, and the message here accounts for about 1.15% of collagen transcripts and 0.14% of overall transcripts [23, 27]. In summary, COL27A1 is the critical gene involved in the differentiation of the somatic ganglion to the spinal column.

## 5. Conclusion

In conclusion, we identified the COL27A1 gene signature based on the GEO database and transcriptome PSCS cohorts. This gene signature was an independent predictive factor for PSCS. Our finding suggested that COL27A1 might contribute to the development of individualized treatment clinically. This study is only a preliminary screening of the PSCS-related hub gene; then, COL27A1 in the PSCS progression and the role of the mechanism is still unknown. Next, we will construct a CS animal model to further understand the mechanism of COL27A1 in the occurrence and development of PSCS.

## Figures and Tables

**Figure 1:** The expression profiling changes of mRNAs in the GSE11854 dataset and GO and KEGG analysis of DEGs. The heat map (a) and volcano plot (b) of DEGs. The bar plots of GO enrichment results of DEGs (c) and the bar plots of KEGG pathway analysis of DEGs (d). DEGs: differentially expressed genes.

RETRACTED

**Figure 2:** DO function analysis. The bar plots of DO analysis results of DEGs (a) and DEG-related DO annotation (b). DEGs: differentially expressed genes.

**Figure 3:** LASSO regression analysis of candidate hub genes. The LASSO analysis of DEGs (a) and 9 candidate hub genes (b). DEGs: differentially expressed genes.

**Figure 4:** Identification of DEGs in patients with PSCS. The heat map (a) and volcano plot (b) of PSCS-related DEGs. DEGs: differentially expressed genes.

**Figure 5:** Functional enrichment analysis of PSCS-related DEGs. The circle plots of GO enrichment results of DEGs (a). The bar plots of BP results (b) and CC results (c) of DEGs. The circle plots of KEGG pathway analysis of DEGs (d). The bar plots of top 20 pathways are shown in (e). DEGs: differentially expressed genes.

**Figure 6:** COL27A1 as the hub gene for PSCS prediction as well as experimental validation. Venn plots of overlapping genes. RT-PCR analysis of COL27A1 mRNA expression in the PSCS group (^∗∗^*P* < 0.05 vs. CON group).

**Table 1:** Inclusion and exclusion criteria.

	Inclusion criteria	Exclusion criteria
PS-CS subjects	Diagnosed PS-CS; obtained informed consent; obtained complete clinical and radiographic data (including X-rays of spinal, CT, and 3D reconstruction and whole spine of MRI)	Informed consent was not obtained; associated with other systemic organic diseases; diagnosed CS-form obstacles (FO) and CS-mixed malformation (MM)
Healthy	No known diseases; obtained informed consent; obtained complete clinical and radiographic data (no spinal deformity using X-rays)	Informed consent was not obtained; patients suffering from an illness

**Table 2:** The top upregulated and downregulated mRNAs in the GSE11854 dataset.

Gene ID	Gene name	Log_2_ fold change	*P* value
Upregulated			
244570_at	LOC101928433	2.288037733	0.000755874
207978_s_at	NR4A3	2.33987635	0.00246423
226709_at	ROBO2	2.3438512	4.45*E* − 05
207850_at	CXCL3	2.396670467	0.000702007
209457_at	DUSP5	2.418294317	2.61*E* − 05
204802_at	RRAD	2.7675236	0.000989502
203407_at	PPL	2.830456133	0.000266057
205266_at	LIF	2.926773717	0.000384075
225016_at	APCDD1	2.991853633	2.38*E* − 05
202768_at	FOSB	5.818043783	0.000608707
Downregulated			
218585_s_at	DTL	-3.675887833	2.04*E* − 06
220651_s_at	MCM10	-3.20875725	3.40*E* − 05
204146_at	RAD51AP1	-3.1408962	0.001056835
229551_x_at	ZNF367	-3.019824967	1.37*E* − 05
1557128_at	FAM111B	-3.0156288	3.13*E* − 05
228281_at	DDIAS	-2.906803233	0.001900307
209832_s_at	CDT1	-2.865265217	2.45*E* − 06
204603_at	EXO1	-2.8420321	0.00013937
203967_at	CDC6	-2.837149017	7.23*E* − 06
205034_at	CCNE2	-2.814359483	9.55*E* − 06

RETRACTED

**Table 3:** The top 10 upregulated and downregulated mRNAs in patients with PSCS.

Gene ID	Gene name	Log_2_ fold change	*P* value
Upregulated			
ENSG00000159063	ALG8	5.108333333	0.00334063
ENSG00000169372	CRADD	5.249	0.008460931
ENSG00000086666	ZFAND6	5.59425	0.005310743
ENSG00000123268	ATF1	5.740083333	0.01453094
ENSG00000042429	MED17	6.16775	0.038970858
ENSG00000171051	FPR1	7.187333333	0.038263095
ENSG00000172322	CLEC12A	9.294166667	0.042669629
ENSG00000132965	ALOX5AP	10.7365	0.015154392
ENSG00000115271	GCA	12.04925	0.026778613
ENSG00000118520	ARG1	14.99491667	0.000598162
Downregulated			
ENSG00000149823	VPS51	-24.99858333	0.037767189
ENSG00000273703	H2BC14	-22.99883333	0.019639801
ENSG00000149591	TAGLN	-22.98425	0.039902194
ENSG00000277075	H2AC8	-17.05541667	0.034354567
ENSG00000120742	SERP1	-16.89908333	0.02256425
ENSG00000158805	ZNF276	-16.20491667	0.027587092
ENSG00000172809	RPL38	-15.6075	0.017643785
ENSG00000197728	RPS26	-14.58275	0.023840796
ENSG00000121060	TRIM25	-14.443	0.027733324
ENSG00000142089	IFITM3	-13.404	0.039033591

**Table 4:** KEGG pathway in patients with PSCS.

Pathway ID	Pathway	*P* value	*Q* value
ko00340	Histidine metabolism	0.008648601	0.08814404
ko04260	Cardiac muscle contraction	0.03252839	0.08814404
ko05410	Hypertrophic cardiomyopathy (HCM)	0.03323526	0.08814404
ko04931	Insulin resistance	0.04028505	0.08814404
ko04670	Leukocyte transendothelial migration	0.04204213	0.08814404
ko04371	Apelin signaling pathway	0.04974778	0.08814404
ko04910	Insulin signaling pathway	0.05184213	0.08814404
ko04261	Adrenergic signaling in cardiomyocytes	0.0539334	0.08814404
ko05414	Dilated cardiomyopathy (DCM)	0.05914811	0.08814404
ko04530	Tight junction	0.06296003	0.08814404
ko04510	Focal adhesion	0.07227287	0.09072276
ko04810	Regulation of actin cytoskeleton	0.07776237	0.09072276
ko05131	Shigellosis	0.0876568	0.09439963
ko01100	Metabolic pathways	0.4628025	0.4628025

## Data Availability

The data used to support the findings of this study are currently under embargo while the research findings are commercialized. Requests for data, 12 months after publication of this article, will be considered by the corresponding author.

## Abbreviations

GEO: Gene Expression Omnibus
DEGs: Differentially expressed genes
GO: Gene Ontology
KEGG: Kyoto Encyclopedia of Genes and Genomes
DO: Disease Ontology
LASSO: Least absolute shrinkage and selection operator
COL27A1: Collagen type XXVII alpha 1 chain
BP: Biological process
CC: Cellular component
MF: Molecular function
TGF-*β*: Transforming growth factor beta 1
CD83: CD83 molecule
SHF: Src homology 2 domain containing F
ORC6: Origin recognition complex subunit 6
GALE: UDP-galactose-4-epimerase
CDT1: Chromatin licensing and DNA replication factor 1
KIRREL3: Kirre-like nephrin family adhesion molecule 3.
